The article "Giant Pseudocyst of the Pancreas: A Case Report" was published in 2022. Journal: Cureus.

# Giant Pseudocyst of the Pancreas: A Case Report

**DOI:** 10.7759/cureus.29456

**Published:** 2022-09-22

**Authors:** Harjit Singh Nalwa, Santh Prakash Lanka, Raul Mederos

**Affiliations:** 1 General Surgery, D.Y. Patil University School of Medicine, Navi Mumbai, IND; 2 General Surgery, Rangaraya Medical College, Kakinada, IND; 3 Surgery, Hialeah Hospital, Hialeah, USA

**Keywords:** pancreatic cyst, huge pseudocyst of the pancreas, cystogastrostomy, pancreas disease, giant pancreatic pseudocyst

## Abstract

Pancreatic cysts are usually asymptomatic over 70% of the time. They can be benign or malignant. Enhanced imaging modalities and increased usage of routine imaging have increased the identification of pancreatic cysts. If symptomatic, abdominal pain or back pain, unexplained weight loss, jaundice, steatorrhea or palpable mass are usually the presenting complaints. Pancreatic cysts are typically assessed by cross-sectional computed tomography (CT) and magnetic resonance imaging (MRI). In this article, we present a case of a 33-year-old female with a recurrent large pancreatic pseudocyst, initially measured 15.8 cm x 14 cm x 14 cm, who was subsequently admitted to our unit and managed successfully. After undergoing diagnostic laparoscopy, exploratory laparotomy, and pancreatic cystogastrostomy, the pseudocyst shrunk to 8 cm x 6 cm over 13 weeks. It is rare to come across a pseudocyst of such large dimensions. Despite its large size, the patient presented with vague abdominal pain as the only chief complaint. The unusual presentation of symptoms and the enormous size of the pseudocyst make this a unique case. Managing giant pancreatic pseudocysts can be complex, as seen in this scenario by the multiple approaches attempted to treat the pseudocyst.

## Introduction

Identification of pancreatic cysts is on the rise due to the enhanced imaging modalities and increased usage of routine imaging. Pancreatic cysts may be a risk factor for developing pancreatic cancer [1]. Pancreatic cysts can be of many types, ranging from benign to malignant [2]. It is essential to obtain a diagnosis as to the etiology of the cyst because more than half of them can be either premalignant or malignant [3]. Almost 15% to 30% of these cysts are pancreatic pseudocysts [4]. They can be single or multiple, with a wide range of clinical manifestations. A pseudocyst with the longest diameter of 10 cm is termed a giant pseudocyst [5], which is increasingly infrequent due to modern treatment options.

A pancreatic pseudocyst is usually diagnosed by ultrasound, computed tomography (CT) scan, or magnetic resonance imaging (MRI). Transabdominal ultrasonography should be utilized as the first step in diagnosing pancreatic pseudocysts. High-resolution endoscopic ultrasound (EUS) detects cystic lesions less than 2 cm in diameter and appears to be of high diagnostic sensitivity. In addition to being an important tool for the diagnosis of pseudocysts, endoscopic retrograde cholangiopancreaticography (ERCP) is equally important for endoscopic therapy [6].

Asymptomatic pseudocysts up to 6 cm in diameter can be safely kept under observation and monitored with recurrent imaging, but larger and symptomatic pseudocysts require intervention [7]. Here, we describe a case of a young female with a very large pseudocyst identified on routine examination during her pregnancy and was recurrent in nature. The patient had to undergo multiple procedures through various approaches for the resolution of the pseudocyst. Only a few cases of giant pancreatic pseudocysts have been documented to date.

## Case presentation

We present a case of a 33-year-old female with a recurrent large pancreatic pseudocyst. The patient was initially found to have a mass two years ago in the left upper quadrant region on examination during the second trimester of her pregnancy, which was identified as a pseudocyst of the pancreas. The patient presented with no complaints of abdominal pain, fever, chills, nausea or vomiting, and no previous history of alcohol consumption. An ultrasound showed the presence of a sizeable septated pancreatic cyst with measurements of 15.8 cm x 14 cm x 14 cm present near the tail of the pancreas with no mural nodules and calcifications, as seen in Figure 1, which was identified as a pseudocyst of the pancreas.

**Figure 1:** Ultrasound of the pancreatic cyst prior to percutaneous drainage. Blue arrows indicate the boundaries of the pancreatic cyst, and white arrows indicate the septations within the pancreatic cyst.

Percutaneous drainage of the pancreatic pseudocyst was performed after an MRI confirmed the presence of the pseudocyst. A follow-up ultrasound 15 days later showed no significant changes in the mass with measurements of 16 cm x 16 cm x 10 cm with septated cystic structure (Figure 2). The patient was later lost to follow-up. However, 21 months later, the patient presented to the clinic complaining of abdominal pain and discomfort. However, she did not report any complaints of nausea, vomiting, early satiety, fever, and chills.

**Figure 2:** Ultrasound one week after percutaneous drainage. Blue arrows highlight the boundaries of the pancreatic cyst.

Referral for endoscopic cystogastrostomy to the Gastroenterology service was made, which turned out to be unsuccessful, leaving us with only a surgical approach with an attempt to remove the pseudocyst completely. If unable to do so, the goal was to perform a cystogastrostomy. Initially, a laparoscopic approach was attempted, which showed the pseudocyst encompassing a third of the abdomen, pushing both the stomach and colon inferiorly. The pseudocyst could not be dissected and separated from the lesser omentum via a laparoscopic approach. At this point, the laparoscopy was converted to open laparotomy with a midline incision extending from the xiphoid process to the umbilicus. Initially, excision of the pseudocyst was attempted, but the pedicle could not be identified. Therefore, a cystogastrostomy was performed rather than excision of the pancreatic pseudocyst, creating an anastomosis between the posterior wall of the stomach and the anterior part of the pseudocyst using an Echelon stapler of size 60. Two small incisions were made, one on the posterior wall of the stomach and another one on the anterior wall of the pseudocyst. Upon doing so, 2.2 L of fluid was drained from the pseudocyst. A sample of the fluid was sent for culture and sensitivity, which turned out to be negative. Then side-to-side anastomosis was created between the posterior wall of the stomach and the anterior wall of the pseudocyst. The anastomosis was noted to be widely patent and with good color and tension-free. 3-0 Vicryl sutures reinforced the anastomosis, and Eviseal was sprayed in the area, ensuring complete hemostasis. The abdomen was irrigated with normal saline and aspirated, with no evidence of bleeding or injury to the intra-abdominal organs. A CT scan of the abdomen without oral contrast was performed on postoperative day 2, which showed a large complex collection of fluid and inflammatory standing with possible debris. The measurements were 8.8 cm x 15.4 cm x 15.8 cm (Figure 3).

**Figure 3:** Non-contrast CT scan of the abdomen on postoperative day 2. Blue arrows point toward the boundaries of the pancreatic cyst, and the cyst is filled with inflammatory debris, which appears as hypodense on the CT scan.

A CT scan of the abdomen with oral contrast was done eight days after the surgery, which showed a mass with measurements of 15 cm in the transverse dimension, 16 cm in the vertical dimension, and 11 cm in the AP dimension (Figure 4). Oral contrast within the mass implies the success of anastomosis between the stomach and the pseudocyst.

**Figure 4:** Oral contrast CT scan of the abdomen on postoperative day 8. Blue arrows point toward the pancreatic cyst, which is markedly reduced in size.

The patient had a follow-up visit at the office three weeks after surgery, and she reported improvement in her symptoms with a CT scan of the abdomen without contrast showing no significant changes (Figure 5). Later, the patient had a follow-up CT scan 13 weeks post-surgery, which showed resolution in size of the pseudocyst to 8 cm x 6 cm (Figures 6, 7).

**Figure 5:** Non-contrast CT scan of the abdomen three weeks post-surgery. Blue arrows highlighting the margins of the pancreatic cyst

 

**Figure 6:** Non-contrast CT scan of the abdomen in a coronal plane three months post-surgery. Blue arrows highlight the boundaries of the pancreatic cyst.

**Figure 7:** Non-contrast CT scan of the abdomen three months post-surgery. Blue arrows highlight the margins of the pancreatic cyst.

## Discussion

According to the Atlanta Symposium, a fluid collection more than 6 to 8 weeks old and surrounded by a wall is defined as a pancreatic pseudocyst [8]. Pancreatic pseudocysts are histopathologically defined as fluid-filled cavities from the pancreas surrounded by a wall of fibrous or inflammatory tissue without an epithelial lining [9]. The Atlanta classification system further subdivides the pancreatic pseudocysts into four entities: (a) acute fluid collection, (b) acute pseudocysts, (c) chronic pseudocysts, and (d) pancreatic abscess [8,10]. Over the years, a significant number of giant pseudocysts have been reported in the medical literature. Bozeman reported the largest recorded pancreatic pseudocyst in 1882, which weighed 10 kg.

Pancreatic cysts are classified into inflammatory fluid collections, non-neoplastic pancreatic cysts, and pancreatic cystic neoplasms. Acute peripancreatic fluid collections, pseudocyst, acute necrotic collections, and walled-off necrosis constitute the inflammatory fluid collections. Non-neoplastic pancreatic cysts include true cysts, retention cysts, mucinous non-neoplastic cysts, and lymphoepithelial cysts. Serous cystic neoplasms, mucinous cystic neoplasms, intrapapillary mucinous neoplasms, and solid pseudopapillary neoplasms are the subtypes of pancreatic cystic neoplasms [11].

Pancreatic pseudocyst is usually a sequela of pancreatitis, which can be caused by numerous etiologies such as alcoholism, biliary stones, and trauma, or could be idiopathic [12]. The highest incidence of pancreatic pseudocysts is likely found in patients with chronic pancreatitis due to alcohol abuse. In a study of 97 patients with pseudocysts, alcohol consumption was the causative factor in 64% of patients with chronic pancreatitis and 26% of patients with acute pancreatitis [13]. More than 70% of pancreatic cysts are asymptomatic when identified. When symptomatic, they present with abdominal or back pain, unexplained weight loss, jaundice, steatorrhea, or palpable mass [3]. The most common manifestations include duodenal or biliary obstruction, vascular occlusion, fistula formation, or digestion of an adjacent vessel resulting in pseudo-aneurysms [14].

Cross-sectional imaging with CT scan and MRI are the mainstay of assessment in pancreatic cysts [1]. Based on the CT imaging findings, pancreatic cystic neoplasms can be eliminated as the cause since the cyst is well-defined and homogenous, and lacks calcifications and mural nodules [15]. Concerning our patient, no duct dilations were noted on imaging, and due to the clear nature of the fluid drained, we excluded retention cysts and mucinous cysts. Apart from the imaging reports of our patient showing septations, the rest of the features, such as homogeneity, presence of internal debris and well-defined wall, all point toward the diagnosis of pancreatic pseudocyst [16].

Biochemical and microbiological analysis of cyst fluid obtained by EUS-guided puncture lacks sensitivity; hence, it is not a reliable tool to diagnose the cause of the pancreatic cyst [17]. In the past, surgical drainage was the only treatment consisting of internal drainage (in the form of cystogastrostomy, cystoduodenostomy, or a Rouen-en-Y cystojejunostomy), external drainage, or excision of the pseudocyst. Today, more advanced treatment options, such as endoscopic drainage and radiological imaging with percutaneous catheter drainage, have become available [15]. However, a randomized controlled trial including 168 patients demonstrated that endoscopic drainage was associated with higher success rates compared to percutaneous drainage (70% vs 31%) with lesser residual collections (21% vs 67%) and lower requirement of surgery in the future (4% vs 11%) [18]. Laparoscopic cystogastrostomy and video-assisted pancreatic necrosectomy have also been successfully used with good outcomes. Some studies have also shown the feasibility of video-assisted necrosectomy as a safer procedure in certain situations for the management of pseudocysts.

Current American College of Gastroenterology guidelines on the management of pancreatic cysts is mentioned in Figure 8 [19]. Intervention for pancreatic pseudocyst is indicated in those patients who present with symptoms such as nausea, vomiting, early satiety, pain, and upper gastrointestinal bleeding. Intervention is also indicated in case of complicated pancreatic pseudocysts (one criterion sufficient) such as gastric or duodenal obstruction, compression of large vessels, stenosis of the common bile duct due to compression, infected pancreatic pseudocysts, hemorrhage into the pseudocyst, or pancreaticopleural fistula. In addition, intervention is indicated in those patients who may be asymptomatic but with a pseudocysts size greater than 5 cm, with the size and morphology remaining unchanged for at least six weeks [6,20,21].

**Figure 8:** American Association of Gastroenterology treatment guidelines for the management of pancreatic cysts. [19] Obtained permission from the original authors EUS, endoscopic ultrasound; FNA, fine needle aspiration; MRI, magnetic resonance imaging; IPMN, intraductal papillary mucinous neoplasm; MCN, mucinous cystic neoplasm

There are only a handful of case studies in literature regarding the management of giant pseudocysts. Behrman et al. concluded that the management of giant pseudocysts was associated with higher morbidity and mortality than the management of small pseudocysts. They suggested external drainage before clinical deterioration [10]. However, there have been reports of large pancreatic pseudocysts treated with laparoscopic cystogastrostomy with good outcomes [22].

A 15-year retrospective analysis conducted in a tertiary hospital in China including 4,379 pancreatitis patients showed that the recurrence rate in pancreatic pseudocyst patients treated with percutaneous drainage was the highest (16.3%) among the three intervention groups. In addition, this study identified that percutaneous drainage was the only risk factor for pancreatic pseudocyst recurrence (OR: 7.812; 95% CI: 3.109-23.072; p = 0.013). This study concluded that a higher recurrence rate is found in pancreatic pseudocyst patients treated with percutaneous drainage compared to endoscopic and surgical interventions [23].

A pancreatic pseudocyst with such large dimensions, as seen in this patient's case, is extremely rare. In addition, the recurrence of the pseudocyst, along with vague abdominal pain as the only presenting complaint despite the large size of the pseudocyst, makes this a unique case. Furthermore, the multiple approaches attempted to treat the pancreatic pseudocyst, in this case, showcase the complexity involved in the management of giant pancreatic pseudocysts.

## Conclusions

We presented a case of a patient with giant recurrent non-neoplastic pancreatic pseudocyst with minimal abdominal discomfort that was diagnosed by imaging. Giant pancreatic pseudocysts are extremely rare, with very few documented case reports. Initial treatment was attempted through endoscopic and laparoscopic approaches, which were unsuccessful. Excision was unsuccessful as the pedicle of the cyst could not be identified. Eventually, a pancreatic cystogastrostomy was successfully carried out through an open approach. We would not recommend percutaneous drainage as the initial mode of treatment, considering the associated recurrence rates. Instead, we would recommend EUS-guided internal drainage as the initial management method of giant pseudocysts. In addition, we recommend early drainage and excision of the pseudocyst before it enlarges to avoid complications during surgery and prevent clinical deterioration. In conclusion, we would like to highlight the mild and vague symptoms the patient experienced despite the enormous size of the pseudocyst, along with the recurrence of the pseudocyst in this case. Furthermore, the complexity of managing the patient with multiple treatment approaches must be highlighted. Cystogastrostomy can be effective in the treatment of giant pancreatic pseudocysts.
